# Bactericidal/Permeability-Increasing Protein Improves Cognitive Impairment in Diabetic Mice *via* Blockade of the LPS-LBP-TLR4 Signaling Pathway

**DOI:** 10.3389/fphys.2020.00718

**Published:** 2021-02-11

**Authors:** Qin Sun, Tingxin Li, Yamei Li, Lingling Wei, Min Zhang, Shaoping Deng

**Affiliations:** ^1^School of Medicine, University of Electronic Science and Technology of China, Chengdu, China; ^2^Health Management Center, Sichuan Academy of Medical Sciences and Sichuan Provincial People’s Hospital, Chengdu, China; ^3^Center of Diabetes Mellitus, Sichuan Academy of Medical Sciences and Sichuan Provincial People’s Hospital, Chengdu, China

**Keywords:** diabetes, cognitive impairment, bactericidal/permeability-increasing protein, lipopolysaccharide-lipopolysacharide-binding protein-toll-like receptor 4 signaling pathway, high-fat diet

## Abstract

Emerging evidence suggests that the bactericidal/permeability-increasing protein (BPI) is involved in the process of cognitive impairment in diabetes. However, its underlying mechanism remains elusive. In this study, we found that BPI affects cognitive impairment due to diabetes through the lipopolysaccharide (LPS)-lipopolysacharide-binding protein (LBP)-toll-like receptor 4 (TLR4) signaling pathway. We examined the expression of BPI, LPS, LBP, CD14, and TLR4 in established mouse models of diabetes induced by high-fat diet (HFD) in combination with streptozotocin (STZ). Diabetic mice were then injected with adeno-associated-virus carrying BPI overexpression vectors and LPS. Fasting blood glucose, plasma insulin, and serum levels of inflammatory factors were examined. Then, glucose tolerance and, insulin resistance tests were used to measure systemic insulin sensitivity. Next, hippocampal tissue injury and cell apoptosis were examined by hematoxylin-eosin (HE) and terminal deoxynucleotidyl transferase-mediated dUTP-biotin nick end labeling (TUNEL) staining. Diabetic mice displayed increased LPS expression and activation of the LPS-CD14-TLR4 signaling pathway. HFD mice following LPS treatment showed significantly increased serum levels of tumor necrosis factor-α (TNF-α), interleukin (IL)-1β, and IL-6, and expressions of Bcl-2-associated X protein (Bax) and Aβ but decreased expression of Bcl-2 in hippocampal tissues, as well as enhanced fasting blood glucose, plasma insulin, glucose tolerance, insulin tolerance, cell apoptosis, aggravated hippocampal tissue injury and, ultimately, cognitive impairment. However, overexpression of BPI was able to rescue the aforementioned phenotypes driven by LPS treatment. Taken together, BPI could potentially provide relief from cognitive impairment in diabetic mice by disrupting the LPS-LBP-TLR4 signaling pathway, underscoring a possible alternative therapeutic strategy against the cognitive impairment associated with diabetes.

## Introduction

Diabetes remains one of the most concerning public health concerns of the twenty-first century in developing countries, due in large part to the lack of accurate monitoring and surveillance (Zimmet et al., 2016). In addition, untimely deaths, medical complications and, financial burdens are on the rise due to the prevalence of undiagnosed diabetes, lack of education about this disease and, insufficient clinical practice standards (Koley et al., 2016). Diabetes has been confirmed to be a driver of disabling vascular complications, new non-vascular complications, and frailty (Sinclair et al., 2015). Patients with diabetes also display a decline in cognitive function, especially with regards to memory, executive functions, and psychomotor efficiency while also having an elevated risk of vascular dementia and Alzheimer’s disease (Pasquier, 2010; Biessels and Despa, 2018). Current treatments include glycemic control, reduction of blood pressure using agents that block the renin-angiotensin system, and control of dyslipidaemia (Harcourt et al., 2013). Better understanding of the relationship between diabetes and cognitive impairment can help improve our management of symptoms and lead to more effective treatment for diabetic patients (Koekkoek et al., 2015).

The bactericidal/permeability-increasing (BPI) protein is an endogenous protein with antimicrobial properties (Zhou et al., 2013, 2014) which acts as a super-antibiotic due to its endotoxin-neutralizing activity (Luo et al., 2012; Qin et al., 2017). Compelling evidence has highlighted a strong link between BPI and diabetes. For example, BPI is significantly lower among patients suffering from type 2 diabetes (T2DM) and it has been found to be correlated negatively with fasting and postload glucose and insulin concentrations (Gubern et al., 2006; Morosky et al., 2016; Wang et al., 2017). Lipopolysaccharide (LPS)-induced increased levels of serum glucose, lactate, and tumor necrosis factor-α (TNF-α) in rats with endotoxemia can be inhibited significantly by simultaneous infusion of BPI (Lin et al., 1994). Moreover, BPI has also been reported to bind to bacteria-derived LPS (Iizasa et al., 2016). LPS is a main component of the outer wall of Gram-negative bacteria (Guo and Chen, 2019). LPS has been found to inhibit the expression of the vitamin D receptor in mononuclear cells of patients with T2DM or diabetic nephropathy uremia (Wu and Cui, 2016). A previous study has also shown that sensitization to LPS is associated with elevated LPS-binding protein (LBP) in animal models (Fang et al., 2013). Recent studies have shown a close relationship between circulating LBP levels and obesity, diabetes, and cardiovascular diseases (Sakura et al., 2017). LBP concentration is noted to be much higher in diabetic patients compared to healthy controls (Gomes et al., 2017). LBPs are important antibacterial innate immunity proteins designed to bind LPS and help present it to cell surface receptors cluster of differentiation 14 (CD14) and toll-like receptor 4 (TLR4; Baron et al., 2016). The transfer of LPS to TLR4-MD2 has been shown to be catalyzed by LBP (Ryu et al., 2017). In addition to its primary role in pathogen recognition, TLR4 is also well known for regulating inflammation (Ma et al., 2015). The transfer of LPS to TLR4-MD2 has been shown to be catalyzed by LBP (Ryu et al., 2017). Expression of TLR4 is increased in streptozotocin (STZ)-induced diabetic mice (Wang et al., 2018). In this study, we investigate the regulatory mechanism of BPI in the LPS-LBP-CD14 signaling pathway associated with cognitive impairment after diabetes, and find a promising clinical therapy for diabetes with cognitive impairment.

## Materials and Methods

### Ethics Statement

The current study was performed with the approval of the Ethics Committee of Sichuan Academy of Medical Sciences and Sichuan Provincial People’s Hospital. Animal experiments adhered strictly to the principle of minimizing the pain, suffering, and discomfort of experimental animals.

### High-Fat Diet/STZ-Induced Mouse Diabetes Model

A total of 120 male specific pathogen-free (SPF) grade C57BL/6J mice (aged 3–4 weeks, weighing 11–14 g) purchased from the Jackson Laboratory for Genomic Medicine (Farmington, Connecticut, USA) were selected for this study. Twelve of them were randomly selected and fed with a normal diet (ND), serving as the control group, and the remaining 108 mice were fed with high-fat diet (HFD)/STZ for diabetes induction as previously reported (Guan et al., 2016). At last, a total of 84 mice were successfully induced. Each mouse was then housed in an SPF animal laboratory with a humidity of 60–65% and a temperature of 22–25°C. After 7 days of adaptive feeding, the mice in the control group were placed on a ND supplemented with 10% calories from fat (TD94149, Harlan Teklad, Indianapolis, IN, USA), and mice in the diabetes group were placed on a HFD supplemented with 45% calories from fat (TD.06415, Harlan Teklad, Indianapolis, IN, USA). After 12 weeks, STZ (45 mg/kg in 0.1 mmol/L sodium citrate, pH 5.5) was intraperitoneally injected into the HFD mice, while the ND-fed mice were injected with the same amount of sodium citrate. After successful model construction, adeno-associated-virus vectors (1 × 10^11^ v.g./100 μl) were injected into the mice in the diabetes group *via* hippocampus once and tail veins twice per week, for a total of 4 weeks. The mice were then divided into seven groups (*n* = 12 per group): HFD (the mice were fed with HFD and injected with STZ), HFD + vehicle (the mice were fed with HFD and injected with the vehicle of LPS), HFD + LPS (the mice were fed with HFD and injected with STZ and LPS), HFD + overexpression negative control (oe-NC; the mice were fed with HFD and injected with STZ and empty vector adeno-associated-virus), HFD + oe-BPI (the mice were fed with HFD and injected with STZ and oe-BPI adeno-associated-virus), HFD + LPS + oe-NC (the mice were fed with HFD and injected with STZ, LPS, and empty vector adeno-associated-virus), and HFD + LPS + oe-BPI (the mice were fed with HFD and injected with STZ, LPS, and oe-BPI adeno-associated-virus). After the successful model induction, the mice were administered 100 μg/kg LPS by intraperitoneal injection for 4 weeks. The mice were given *ad libitum* access to water and housed in a room under a 12-h light/dark cycle. After 72 h of STZ injection, the blood samples of tail veins were taken for blood glucose analysis to confirm successful model construction. The mice with blood glucose level > 11.1 mmol/L were considered to be diabetic mice. After LPS or adeno-associated-virus injections, the mice were further raised for 7 weeks. At the end of the experiment, six mice were randomly selected from each group and euthanized *via* anesthesia by 1% pentobarbital sodium injection. Then hippocampal tissues of mice were harvested for subsequent experiments.

### Determination of LPS Plasma Level

The LPS plasma level was determined using a Limulus amebocyte extract kit according to the manufacturer’s instructions (LAL kit; Cambrex BioScience, Walkersville, MD, USA).

### Reverse Transcription Quantitative Polymerase Chain Reaction

Total RNA from hippocampal tissues of mice in each group was extracted using TRIzol (Sigma-Aldrich, St. Louis, MO, USA). The extracted RNA was then reversely transcribed into complementary DNA (cDNA) using the PrimeScript™ RT Reagent Kit (TaKaRa, Tokyo, Japan). Then, reverse transcription quantitative polymerase chain reaction (RT-qPCR) was carried out in accordance with the instructions of the SYBR® Premix Ex Taq™ II (Tli RNaseH Plus) kit (TaKaRa, Tokyo, Japan). The product was then amplified using the Thermal Cycler Dice Real Time System (TP800, TaKaRa, Tokyo, Japan). Triplicate wells were set in each group. The gene specific primers were synthesized by Shanghai Sangon Biotech Company (Shanghai, China), with the sequences shown in Table 1. With glyceraldehyde-3-phosphate dehydrogenase (GAPDH) used as an internal reference, the expression of target genes was calculated using the 2^^(-ΔΔCT)^ method.

**Table 1:** Primer sequences for RT-qPCR.

Gene	Primer sequences
BPI	F: 5'-GGTAAGAAGGAAAACAAATGCC-3'
	R: 5'-AACCACCTGCTGCCAA-3'
GAPDH	F: 5'-GCAAATTCAACGGCACAGTCAA-3'
	R: 5'-AAGACACCAGTAGACTCCACGACAT-3'

RT-qPCR, reverse transcription quantitative polymerase chain reaction; BPI, bactericidal/permeability-increasing protein; GAPDH, glyceraldehyde-3-phosphate dehydrogenase; F, forward; R, reverse.

### Western Blot Analysis

The hippocampal tissues of each group were collected and washed with phosphate buffer saline (PBS). Then the tissues were incubated with protein lysis reagents containing protease and alkaline phosphatase inhibitor (C0481, Sigma-Aldrich, St. Louis, MO, USA) at 4°C for 30 min. The cell lysate was collected into a 1.5 ml Eppendorf tube, and centrifuged at 10,000 rpm for 15 min, followed by supernatant collection. The protein concentration was measured using the Bradford method according to the kit instructions (TaKaRa Bradford Protein Assay Kit, No. T9310A, TaKaRa, Tokyo, Japan). Next, 20 μg of protein was separated with 10% sodium dodecyl sulfate-polyacrylamide gel electrophoresis (SDS-PAGE) and transferred to a polyvinylidene fluoride (PVDF) membrane. Then, the membrane was blocked using 5% skim milk powder for 1 h and probed overnight at 4°C with rabbit monoclonal antibodies against B-cell lymphoma-2 (Bcl2; ab182858, 1:2,000), Bcl-2-associated X protein (Bax; ab32503, 1:1,000), CD14 (ab221678, 1:1,000), TLR4 (ab13556, 1:500), nuclear factor-κB (NF-κB) p65 (ab16502, 1:2,000), and β-actin (ab124964, 1:10,000). The aforementioned antibodies were purchased from Abcam Inc. (Cambridge, UK). After three washes with Tris-buffered saline with Tween 20 (TBST) three times, the membrane was treated with horseradish peroxidase-labeled secondary goat anti-rabbit (ab205718, 1:2,000) and incubated for 1 h at room temperature. Then, the samples were washed six times with TBST. The immuno-complexes on the membrane were visualized using enhanced chemiluminescence (ECL) reagent, and luminosity of the band was quantified using the ImageJ analysis system. The ratio of the gray value of our protein of interest to that of β-actin was representative of the relative expression.

### Determination of Fasting Blood Glucose and Plasma Insulin

The remaining six mice in each group were fasted overnight 1 week before the end of the experiment. The blood was taken from the tail veins of mice for blood glucose measurement using an Accu-Check Advantage glucometer and blood glucose test strips (Roche Diagnostics GmbH, Mannheim, Germany). According to the manufacturer’s instructions, levels of insulin in plasma were determined using an insulin enzyme-linked immunosorbent assay (ELISA) kit (Linco Research Inc., St Charles, Missouri, USA).

### Enzyme-Linked Immunosorbent Assay

The levels of TNF-α (ab208348, Abcam Inc., Cambridge, UK), interleukin (IL)-1β (ab100704, Abcam Inc., Cambridge, UK), and IL-6 (ab100712, Abcam Inc., Cambridge, UK) in serum of mice in each group were determined according to the manufacturer’s instructions of the ELISA kit (Linco Research Inc., St Charles, Missouri, USA).

### Glucose Tolerance and Insulin Tolerance Tests

One week before the end of the experiment, the remaining six mice in each group were fasted overnight before the glucose tolerance test. Mice were injected intraperitoneally with glucose at a dose of 1.5 g/kg body weight. The blood was taken from the mouse tail vein at 0, 25, 50, 75, 100, and 125 mins, and blood glucose levels were measured. Mice were fasted overnight before the insulin resistance test. Mice were injected intraperitoneally with 0.75 IU/kg insulin. The tail vein blood was taken at 0, 25, 50, 75, 100, and 125 mins, respectively, and blood glucose levels were measured. The insulin resistance index was calculated based on the measured fasting blood glucose and fasting insulin levels: HOMA insulin resistance index (HOMA-IRI) = fasting blood glucose × fasting insulin/22.5.

### Terminal Deoxynucleotidyl Transferase-Mediated dUTP-Biotin Nick End Labeling Staining

Cell apoptosis in mouse hippocampal tissues was measured using terminal deoxynucleotidyl transferase-mediated dUTP-biotin nick end labeling (TUNEL). In short, the hippocampal tissues were fixed with neutral formaldehyde, dehydrated, embedded in paraffin, and cut into sections. The tissue sections were then dewaxed twice with xylene for 5 min, and rehydrated with gradient ethanol (100, 95, 90, 80, and 70%). Following the instructions of the TUNEL kit (Roche, Basel, Switzerland), 50 μl of TUNEL reaction solution (the ratio of enzyme concentration solution and labeling solution was 1:9) was added to the sections for 50 min. Then, 50 μl of transformant-POD was added to the sections and incubated at 37°C for 30 min. Afterward, a total of 100 μl of diaminobenzidine (DAB) working solution was added and incubated for 10 min to develop the sections. The sections were subsequently counterstained with hematoxylin for 3 s and then sealed with neutral gum. The staining results were finally observed under a high-power microscope. The apoptotic cells were finally counted in five randomly selected fields from each group, and the apoptosis rate was calculated using the formula: apoptosis rate = (apoptotic cells/total cells) × 100%.

### Hematoxylin-Eosin Staining

The mouse hippocampal tissues were fixed with formaldehyde, dehydrated conventionally using gradient alcohol (70, 80, 90, 95, 100%, respectively; 5 min/time), cleared twice with xylene (10 min/time), immersed in wax, and embedded into paraffin. Tissues were then sliced continuously at a thickness of 4 μm. The sections were then heated at 60°C for 1 h, de-paraffinized using xylene, and dehydrated with gradient ethanol, followed by washing under tap water. Following that, the sections were stained with hematoxylin for 10 min, immersed in 1% hydrochloric acid alcohol for 20 s, washed with 1% ammonia water for 30 s, stained with eosin for 3 min, dehydrated with gradient ethanol (2 min/time), and rinsed twice using xylene (5 min/time). Next, the sections were sealed with neutral gum, and observed under a 40-fold optical microscope (BX41, Olympus, Tokyo, Japan).

### Morris Water Maze

One week before the end of the experiment, the remaining six mice in each group were subjected to learning and memory ability tests using the Morris water maze experiment. The labyrinth pool had a diameter of 150 cm and a height of 60 cm. The four water inlet points marked on the wall divided the pool into four quadrants, one of which was placed on a platform 1 cm below the water surface. The test comprised of navigation test and space exploration test. The navigation test was conducted to measure the learning and memory ability of mice. Briefly, the mice were allowed to swim freely for 2 min before the day of training, and the platform was higher than the water surface. Formal training lasted 5 consecutive days (4 times/day) and the duration required for mice to find and climb the platform (escape latency) was recorded each time from different position in water. If the mice did not find a platform within 60 s, the mice were assigned to the platform with the escape latency of 60 s. The space exploration experiment was used to evaluate the ability of mice to maintain the memory of finding the platform space after learning. On the fifth day, the platform was removed and the first quadrant was selected. The trajectories of the mice within 60 s and the time spent in each quadrant were recorded and calculated. The percentage of time that mice spent on the platform to that of mice swimming in the pool was calculated by the meandering winding magnetometer (MWM) motion detection software (Actimetrics software, Evanston, I.L, USA).

### Statistical Analysis

All data were analyzed using the SPSS 21.0 statistical software (IBM Corp., Armonk, NY, USA). Measurement data were expressed as mean ± SD. Comparison between two groups was conducted using independent sample *t*-test. Comparisons among multiple groups were conducted using one-way ANOVA followed by a Tukey’s *post hoc* test. The glucose levels of mice at different time points were analyzed using repeated measures ANOVA and the area under the curve was calculated using a software. A value of *p* < 0.05 was considered to be indicative of statistical significance.

## Results

### LPS Overexpression Activates the TLR4 Signaling Pathway in Mice With Diabetes

To study the relevant factors for diabetes induced cognitive impairment, HFD and STZ were used to construct a mouse model of diabetes. To confirm successful induction, the blood glucose level of the mice was measured and the results showed that the blood glucose level of HFD mice was significantly higher than that of the ND-fed mice (Figure 1A). Next, we performed a Morris water maze experiment which showed that the latency time of HFD mice was significantly longer than that of ND-fed mice, while the time HFD mice spent on the platform quadrants and the number of platform crossings was significantly reduced (Figures 1B–D). These results confirm that diabetes induction leads to cognitive impairment in mice. Subsequently, the levels of LPS and LBP in the blood and, the expression of CD14, TLR4, and NF-κB signaling pathway-related factors were examined in mouse hippocampal tissues. The results show significantly increased serum levels of LPS and LBP in mice fed with HFD in addition to elevated expression of CD14 and TLR4 proteins in hippocampal tissues as well as increased nuclear expression of NF-κB p65 compared with mice fed with ND (Figures 1E,F). These results suggested elevated LPS and activation of innate signaling pathways through CD14 and TLR4 in our mouse model of diabetes.

**Figure 1:** Increased lipopolysaccharide (LPS) expression and activated LPS/CD14/toll-like receptor 4 (TLR4) signaling pathway in diabetic mice. **(A)** Fasting blood glucose level of mice in each group. **(B)** The latency time of mice in each group tested by the Morris water maze experiment. **(C)** The time ratio of mice in each group staying on the platform quadrant tested by Morris water maze experiments. **(D)** The time of mice in each group crossing the target platform quadrant. **(E)** The levels of LPS and LBP in the plasma of mice from each group. **(F)** Serum levels of CD14, TLR4, and NF-κB p65 expression in hippocampal tissues of mice in each group. ^*^p < 0.05 vs. the mice fed with normal diet (ND). The results were measurement data and expressed as mean ± standard deviation. Data between two groups were compared by independent sample *t*-test.

### Exogenous LPS Promoted Inflammation, Insulin Resistance, and Cognitive Impairment in Diabetic Mice

We then aimed to further confirm the role of LPS in diabetic mice with cognitive impairment by assessing the level of inflammatory cytokines in the blood. The serum levels of TNF-α, IL-1β, and IL-6 were indeed increased compared with that in the mice fed with ND and the HFD mice injected with vehicle of LPS (Figure 2A). This data indicated that treatment with HFD and STZ could promote an inflammatory response in mice, while the addition of LPS could further increase the inflammatory response in HFD mice. As depicted in Figure 2B, the expression of Bax and Aβ was significantly increased while Bcl-2 expression was significantly decreased in the hippocampal tissues of the HFD-fed mice and the HFD-fed mice injected with LPS compared with that of the ND-fed mice and the HFD-fed mice injected with vehicle of LPS. Additionally, as depicted in Figures 2C–H, HFD-fed mice and the HFD-fed mice injected with LPS exhibited elevated fasting blood glucose levels, plasma insulin, glucose tolerance, and insulin resistance when compared with the ND-fed mice and the HFD-fed mice injected with vehicle. Compared to mice fed with ND and HFD-fed mice injected with vehicle, HFD-fed mice and HFD-fed mice following LPS treatment exhibited numerous damaged neurons in the hippocampal CA1 region, presenting indistinct cell boundaries, with small darkened and shrunken nuclei (Long et al., 2020). In addition, the results of HE staining showed that the hippocampal neurons of ND-fed mice were arranged compactly, while the neurons of HFD-fed mice were dispersed. Further analysis revealed a decline in the number of hippocampal neurons in HFD-fed mice, particularly in HFD-fed mice following LPS treatment. In contrast, ND-fed mice demonstrated only minimal morphological changes (Figure 2I). Furthermore, TUNEL staining analysis revealed that the number of the apoptotic neurons in the CA1 zone was much higher in HFD-fed mice and HFD-fed mice treated with LPS than in ND-fed mice and HFD-fed mice treated with vehicle (Figure 2J; Zhang et al., 2020). The results from HE (Figure 2I) and TUNEL (Figure 2K) staining revealed greater tissue damage and a significantly increased rate of apoptosis in HFD-fed mice and HFD-fed mice treated with LPS as compared with ND-fed mice and HFD-fed mice treated with vehicle. Furthermore, the results of the Morris water maze experiment (Figures 2L–N) showed that the HFD-fed mice injected with LPS exhibited a relatively longer latency time and shorter time spent on the platform quadrant residence, as well as less time crossing the platform than the HFD-fed mice injected with vehicle. These results suggested that exogenous LPS promoted inflammation, insulin resistance, and cognitive impairment in diabetic mice.

**Figure 2:** Inflammation, insulin resistance, and cognitive impairment are promoted by exogenous LPS in diabetic mice. **(A)** Serum levels of inflammatory factors of mice in each group. **(B)** Western blot analysis of Bcl-2-associated X protein (Bax), Aβ, and Bcl-2 proteins in hippocampal tissues of mice in each group. **(C)** The fasting blood glucose of mice in each group. **(D)** Fasting insulin content of mice in each group. **(E)** Blood glucose levels of mice in each group analyzed by a glucose tolerance test. **(F)** The area under the curve (AUC) corresponding to **E**. **(G)** Blood glucose of mice in each group analyzed by insulin resistance test. **(H)** The AUC corresponding to the **G**. **(I)** HE staining of the pathological tissues of the hippocampal tissues of each group (400×). **(J,K)** Cell apoptosis in hippocampal tissues of mice in each group measured by TUNEL staining (400×). **(L)** The latency of mice in each group examined by the Morris water maze experiment. **(M)** The time ratio of mice in each group staying in the quadrant of the platform. **(N)** Times that the mice in each group crossed the target platform quadrant. In panel **(A–K)**, ^*^p < 0.05 vs. the mice fed with ND. ^#^*p* < 0.05 vs. the HFD mice injected with vehicle of LPS. In panel **(L–N)**, ^*^p < 0.05 vs. the HFD mice injected with vehicle of LPS. The results were measurement data and expressed as mean ± standard deviation. Data among multiple groups were compared by one-way ANOVA, followed by Tukey’s *post hoc* tests. *N* = 6 for mice following each treatment.

### Overexpression of BPI Inhibited the LPS-CD14-TLR4 Signaling Pathway, Thereby Blocking NF-κB Signaling

It is reported that BPI has a chemical structure similar to that of LBP. Although it is not a receptor of LPS, BPI can bind to LPS and its binding ability is 20 times that of LBP and LPS. The competitive binding of BPI to LPS with LBP can prevent the inflammatory response caused by the binding of LPS and LBP. Previous studies have shown that 2 ng/ml of BPI can completely inhibit LPS activity. To investigate whether BPI could regulate the amount of LPS leading to excessive inflammation and cognitive impairment in the mouse model of diabetes, we silenced BPI in mice by using an adeno-associated-virus vector. First, we used RT-qPCR (Figure 3A) to determine baseline differences in BPI mRNA expression between HFD-fed and mice fed with ND, which revealed that diabetic mice had significantly reduced expression of BPI. Next, compared with the HFD-fed mice injected with oe-NC, the expression of BPI was increased in hippocampal tissues of HFD-fed mice injected with oe-BPI. In addition, the expression of BPI was increased in the hippocampal tissues of the HFD mice injected with LPS and oe-BPI compared with the HFD mice injected with LPS and oe-NC. Moreover, as displayed in Figure 3B, compared with the HFD mice injected with oe-NC, the expression of CD14 and TLR4 was decreased in hippocampal tissues of the HFD mice injected with oe-BPI, in addition to reduced NF-κB p65 expression observed in the nuclei of hippocampal tissues. A similar trend for the aforementioned factors was noted in the HFD mice injected with LPS and oe-BPI in comparison to HFD mice injected with LPS and oe-NC. These results suggested that overexpression of BPI inhibited the LPS-CD14-TLR4 signaling pathway, which in turn reduced activation of the NF-κB signaling pathway.

**Figure 3:** Forced BPI expression disrupts the LPS-CD14-TLR4 signaling pathway and then inhibits the NF-κB signaling pathway. **(A)** The expression of BPI in the hippocampal tissues of mice in each group examined using reverse transcription quantitative polymerase chain reaction (RT-qPCR). **(B)** Western blot analysis of CD14, TLR4, and NF-κB p65 proteins in hippocampal tissues of mice in each group. ^&^*p* < 0.05 vs. mice fed with ND. ^*^p < 0.05 vs. HFD mice injected with oe-NC. ^#^*p* < 0.05 vs. HFD mice injected with LPS and oe-NC. The results were measurement data and expressed as mean ± standard deviation. Data between two groups were compared by independent sample *t*-test.

### Overexpression of BPI Reduced Inflammation, Insulin Resistance and, Cognitive Impairment in Diabetic Mice

In light of our findings, the effects of BPI overexpression on inflammation, insulin resistance, and cognitive impairment in diabetic mice were further investigated. The serum levels of inflammatory cytokines TNF-α, IL-1β, and IL-6 were determined by standard ELISA. Compared with HFD mice injected with oe-NC, serum levels of these cytokines were decreased in HFD mice injected with oe-BPI. In comparison with HFD mice injected with LPS and oe-NC, the serum levels of TNF-α, IL-1β, and IL-6 were also reduced in the HFD mice injected with LPS and oe-BPI (Figure 4A). These results suggested that overexpression of BPI inhibited the inflammatory response in mice. Next, we noticed a significant decline in the expression of Bax and Aβ, while Bcl-2 expression was increased in hippocampal tissues of HFD mice injected with oe-BPI compared to HFD mice injected with oe-NC (Figure 4B). Compared with HFD mice injected with LPS and oe-NC, the expression of Bax and Aβ was decreased, while the expression of Bcl-2 was increased in hippocampal tissues of the HFD mice injected with LPS and oe-BPI. Figures 4C–H show a downward trend in the fasting blood glucose, plasma insulin, glucose tolerance, and insulin tolerance in the HFD mice injected with oe-BPI, compared to the HFD mice injected with oe-NC. The HFD mice injected with LPS and oe-BPI mice had significantly lower fasting blood glucose, plasma insulin, glucose tolerance, and insulin resistance than the HFD mice injected with LPS and oe-NC. The results of HE and TUNEL staining revealed that the HFD mice injected with oe-BPI had a lower degree of hippocampal tissues damage and apoptosis rate compared with the HFD mice injected with oe-NC (Figures 4I–K). A similar trend for the aforementioned factors was seen in HFD mice injected with LPS and oe-BPI compared to HFD mice injected with LPS and oe-NC. The results of the Morris water maze experiment (Figures 4L–N) showed that the HFD mice injected with oe-BPI or with LPS and oe-BPI had a relatively shorter latency time, longer original platform quadrant residence time, and more times of platform crossings compared with HFD mice injected with oe-NC or with LPS and oe-NC. Taken together, this data suggest that overexpression of BPI reduces inflammation, insulin resistance, and cognitive impairment in diabetic mice.

**Figure 4:** Inflammation, insulin resistance, and cognitive impairment are inhibited following BPI upregulation in diabetic mice. **(A)** Serum levels of inflammatory factors of mice in each group detected by ELISA. **(B)** Western blot analysis of Bax, Aβ, and Bcl-2 proteins in hippocampal tissues of mice in each group. **(C)** Determination of fasting blood glucose levels of mice in each group. **(D)** Quantitation of fasting insulin amount of mice in each group. **(E)** Blood glucose levels of mice in each group using the glucose tolerance test. **(F)** The AUC corresponding to **E**. **(G)** Blood glucose levels of mice in each group using the insulin resistance test. **(H)** The AUC corresponding to the **G**. **(I)** HE staining of the hippocampal tissues of mice in each group (400×). **(J)** Cell apoptosis in the hippocampal tissues of mice in each group detected using TUNEL staining (400×). **(K)** The statistical analysis chart corresponding to **J**. **(L)** The latency of mice in each group determined by Morris water maze. **(M)** The ratio of time that mice in each group staying in the quadrant of the platform. **(N)** The number of mice in each group passing the target platform quadrant. ^*^p < 0.05 vs. the HFD mice injected with oe-NC. ^#^*p* < 0.05 vs. the HFD mice injected with LPS and oe-NC. The results were measurement data and expressed as mean ± standard deviation. Data between two groups were compared by independent sample *t*-test.

## Discussion

The rapid growth of diabetes cases comes with a high economic burden for patients and their families (Jing et al., 2019). In addition to more well-known symptoms, diabetic patients are also at a higher risk of developing cognitive impairments (Albai et al., 2019). In this study, we constructed an HFD/STZ-induced mouse model of diabetes to clarify the possible roles of BPI in cognitive impairment *via* the LPS-LBP-TLR4 signaling pathway (Figure 5).

**Figure 5:** Diagram depicting a potential mechanism of interactions. BPI can alleviate cognitive impairment in diabetic mice by blocking the LPS-LBP-TLR4 signaling pathway. LPS was overexpressed and BPI was poorly expressed in diabetic mice with cognitive impairment. Exogenous LPS promotes inflammation, insulin resistance, and cognitive impairment in diabetic mice. Overexpression of BPI inhibited the LPS-LBP-TLR4 signaling pathway, thereby suppressing the NF-κB signaling pathway and ultimately reducing inflammation, insulin resistance, and cognitive impairment in diabetic mice.

Our initial observations revealed that LPS was overexpressed which resulted in a hyperactive LPS-CD14-TLR4 signaling pathway in our diabetic mice cohort. Our findings are consistent with previously reported increased levels of LPS in T2DM in humans (Jayashree et al., 2014). Moreover, the expression of CD14 is significantly upregulated in patients with impaired glucose tolerance (Terasawa et al., 2015). Another study suggested that the level of CD14 is much higher in patients with diabetes than in healthy volunteers (Stulc et al., 2014). In addition, the mRNA expression of TLR4 has been increased in patients with T2DM (Taha et al., 2018).

Another key observation from the current study was that exogenous LPS promoted inflammation, cell apoptosis, insulin resistance, and cognitive impairment in diabetic mice. Consistent with our findings, overexpression of LPS has been documented to promote the expression of inflammatory cytokines in the brain tissue and inhibit mitochondrial function (Haj-Mirzaian et al., 2019). It has been reported that LPS initiates inflammation, weight gain, and T2DM (Monte et al., 2012). LPS also stimulates the release of IL-6, IL-8, and TNF-α in the supernatants of RAW 264.7 cells in propofol-based anesthesia (Jia et al., 2017). Mechanically, Bcl-2 protein plays an important role in the regulation of cell apoptosis by forming heterodimer and self-dimer with Bax. Specifically, when Bcl-2 protein is inhibited, the formed heterodimer with Bax is reduced, leading to apoptosis. When Bcl-2 protein is overexpressed, the formed heterodimer with Bax is increased, attenuating cell apoptosis. Thus, the balance between Bcl-2 and Bax proteins in the cell death checkpoint signal determines cell survival or apoptosis (Stevens and Oltean, 2019). Low-grade inflammation induced by LPS causes central insulin resistance in obesity (Rorato et al., 2017). Following treatment with LPS, the expression of Bcl-2 is deceased while the expression of Bax is increased, which was shown to inhibit the apoptosis of endometrial cell and benefit embryo implantation (Wang et al., 2016). LPS has been found to cause neuronal PC12 cell death by elevating the expression of pro-apoptotic Bax and increasing the Bax/Bcl-2 ratio (Sharifi et al., 2010). Furthermore, LPS reduces the expression of Bcl-2 while enhancing the expression of Bax and caspase-3, thus inducing apoptosis of STC-1 cells, which may be responsible for the reduced secretion of glucagon-like peptide 1 (GLP-1) well-known for its anti-diabetic activity (Lei et al., 2013). Aβ is known as a causative factor for Alzheimer’s disease and induces neuronal loss through activation of apoptotic pathways (Lei and Renyuan, 2018). Meanwhile, the upregulation of Aβ1–42 is accompanied by an increase in caspase-3 and Bax levels and a decrease in Bcl-2 level in systemic LPS-injected mouse brains (Chen et al., 2017). LPS is not only responsible for memory loss, but also for the increase in the levels of Aβ, nitric oxide, and glutamate in the brain (Ekladious and El Sayed, 2019). Thus, LPS likely acts as a driver of accelerated inflammation, cell apoptosis, insulin resistance, and cognitive impairment in diabetic mice.

Additionally, we found that upregulated BPI could bind to LPS and disturb the inflammation caused by the combination of LBP and LPS. In support of our findings, recent studies show that BPI binding to LPS plays a critical role in the immune system of mammals (Iizasa et al., 2016). Moreover, BPI is known to possess anti-inflammatory properties through its LPS neutralizing activity (Yao et al., 2015). In addition, the results of our study showed that overexpression of BPI inhibited the LPS-CD14-TLR4 signaling pathway, thereby inactivating the NF-κB signaling pathway. BPI binds to LPS leading to disrupted NF-κB signaling exerted by LPS *via* blockade of the TLR4 responses in an extrinsic mode (Azuma et al., 2007). Moreover, BPI and CD14 and their effects have been investigated in hematopoietic cells (Guinan et al., 2014).

Another key finding was that overexpression of BPI in diabetic mice reduced inflammation, insulin resistance, and cognitive impairment *in vivo*. Previous work has reported the anti-inflammatory effect of BPI induced by Gram-negative bacteria (Balakrishnan et al., 2016). Moreover, BPI has been known to be sensitive to insulin in the immune system (Gubern et al., 2006). The bovine full-length BPI or BPI714 can decrease the expression of IL-8, IL-1β, TNF-α, and NF-κB-2 and either bovine BPI or BPI714 can inhibit LPS-stimulated immune response, which shows that BPI/LPS-neutralizing activity has an antibacterial function (Yao et al., 2015). To the best of our knowledge, however, few studies looked at the impact of BPI overexpression on cognitive impairment in diabetes.

Overall, our study showed that when LPS is introduced in diabetic mice, it promotes inflammation, insulin resistance, and cognitive impairment. However, BPI is able to rescue these effects by binding to LPS and reducing the inflammation caused by presentation through LBP. In addition, overexpression of BPI is able to inhibit the NF-κB signaling pathway to improve cognitive impairment induced by diabetes through inhibition of the LPS-CD14-TLR4 signaling pathway. These findings may enable the development of new therapeutic strategies for the prevention and treatment of cognitive impairment in diabetes. However, further *in vitro* studies are still required to elucidate the specific mechanism of the LPS-CD14-TLR4 network involved in cognitive impairment associated with diabetes.

## Data Availability Statement

The raw data supporting the conclusions of this article will be made available by the authors, without undue reservation, to any qualified researcher.

## Ethics Statement

The current study was performed with the approval of the Ethics Committee of Sichuan Academy of Medical Sciences and Sichuan Provincial People’s Hospital. The animal experiment strictly adhered to the principle to minimize the pain, suffering, and discomfort to experimental animals.

## Author Contributions

QS, MZ, and SD designed the study. YL and QS collated the data, carried out data analyses, and produced the initial draft of the manuscript. TL, LW, and QS contributed to drafting the manuscript. All authors have read and approved the final submitted manuscript.

### Conflict of Interest

The authors declare that the research was conducted in the absence of any commercial or financial relationships that could be construed as a potential conflict of interest.
